# Liraglutide Alleviates Diabetic Atherosclerosis through Regulating Calcification of Vascular Smooth Muscle Cells

**DOI:** 10.1155/2022/5013622

**Published:** 2022-04-25

**Authors:** Li-Li Shi, Ming Hao, Zhou-Yun Jin, Gui-Fang Peng, Ying-Ying Tang, Hong-Yu Kuang

**Affiliations:** ^1^Department of Cadre Ward, The First Affiliated Hospital of Harbin Medical University, Harbin 150081, China; ^2^Department of Endocrinology, The First Affiliated Hospital of Harbin Medical University, Harbin 150081, China; ^3^Department of Endocrinology, The Heilongjiang Provincial Hospital, Harbin 150001, China

## Abstract

**Background:**

Diabetes mellitus (DM) is a group of metabolic diseases characterized by hyperglycemia, which can induce the development of atherosclerosis (AS). Calcification of vascular smooth muscle cells (VSMCs) exerts an important role in the process of AS. In this study, the effects of liraglutide (LIRA) on VSMC under high-glucose condition and its mechanism were explored.

**Method:**

After VSMC was treated by high glucose with or without LIRA *in vitro*, the alkaline phosphatase (ALP) activity was measured by the detection kit, osteogenic marker protein expression was detected by Western blotting, and calcification was determined by alizarin red staining. Subsequently, the DM rat model was established and the ALP activity, calcification, and osteogenic marker proteins were determined *in vivo*. Immunohistochemical (IHC) staining and hematoxylin-eosin staining were performed on the thoracic aorta of DM rats.

**Result:**

The positive rate of SM*α*-actin expression in the DM + AS group was significantly lower than that in control rats, but LIRA administration increased the positive rate in the model. The expression of Cbf*α*-1 and OPN in the DM + AS group was significantly higher than that in the control group, while it was decreased after treatment of LIRA. The ALP activity and calcium content were increased in DM + AS rats, and the treatment of LIRA decreased the phenotypes in the rats, so as to delay the progression of AS in DM rats. Meanwhile, LIRA inhibited the ALP activity, upregulated SM-*α* expression, and downregulated expression of OPN and Cbf*α*-1 in VSMC under high-glucose (HG) conditions. Mechanically, HG-enhanced ALP activity, AKT, and ERK phosphorylation were inhibited by LIRA, PI3K antagonist LY294002, or ERK1/2 antagonist PD98059, in which cotreatment of LIRA with LY294002 and PD98059 could further enhance the effect of LIRA on VSMC, and GLP-1R antagonists reversed the phenotypes in the model. LIRA blocked the osteogenic transformation of VSMC through PI3K and ERK1/2 signaling pathways, which can be reversed by GLP-1R antagonists.

**Conclusion:**

LIRA inhibited the abnormalities in VSMC calcification mediated by the GLP-1R, which was related to PI3K/Akt and ERK1/2 MAPK pathways. Therefore, the prospect and significance of LIRA in the treatment of DM complicated with AS were clarified.

## 1. Introduction

Diabetes mellitus (DM) has become a rising epidemic that seriously threatens human health and life. The harm of diabetes to human health mainly comes from the concurrent damage of many organs, especially cardiovascular diseases, such as atherosclerosis (AS) [1]. It has been demonstrated that hyperglycemia can lead to AS through a variety of mechanisms, including the functional regulation of vascular smooth muscle cells (VSMC). Notably, hyperglycemia not only promotes the proliferation and migration of VSMC [2] but also induces osteogenic changes of VSMC, which is one of the main causes of vascular calcification [3]. More importantly, it is well known that vascular calcification is an important pathological process and manifestation of AS [4]. Although traditional hypoglycemic drugs such as biguanides, sulfonylureas, and insulin are capable of alleviating AS [5], they do not provide any guidance. Moreover, long-term application of sulfonylureas and insulin could induce obesity and further increase the risk of cardiovascular disease [6]. Although the mechanistic study has shown that several signaling pathways are involved in the regulation of VSMC calcification in DM combined with AS, such as phosphatidylinositol-4-diphosphate 3-kinase (PI3K)/protein kinase B (AKT) and the ERK1/2 MAPK signaling pathway [7, 8], no targeted therapy has been developed till now. Therefore, inhibiting migration, proliferation, and especially calcification of VSMC could be a promising strategy for the treatment of DM complicated with AS.

Glucagon-like peptide-1 (GLP-1) is an important regulator of glucose metabolism [9]. The GLP-1 receptor (GLP-1R) was expressed on the surface of aortic smooth muscle cells in both humans and rats. Accumulating evidence showed that GLP-1 could stimulate insulin secretion in a glucose-dependent manner, reduce gastric emptying, inhibit food intake, and increase natriuresis [10]. Therefore, after some biomedical modifications for achieving enhanced therapeutic efficiency and sustained effects, GLP-1R agonists have been widely used in the clinical treatment of type 2 diabetes mellitus (T2DM) as well as clinical evaluation of obesity [11]. Moreover, liraglutide (LIRA), which is a synthetic analogue of GLP-1, has also been commonly used in the treatment of DM and obesity [12]. On the other hand, besides the application of GLP-1/GLP-1R in treating DM, recent studies revealed the significant cardio- and neuroprotective effects of GLP-1 [13]. It has been reported that LIRA reduces AS in T2DM rats by targeting ER-associated macrophage-derived macrovesicle production [14]. LIRA represses AS by regulating inflammatory pathways in ApoE^−/−^ mice [15]. LIRA inhibits AS by modulating proinflammatory mediators and immune cell phenotypes in apolipoprotein E-deficient mice [16]. However, till now, the mechanism of the cardioprotective effects of GLP-1R agonists or GLP-1 analogue such as LIRA is rarely reported and remains largely unknown. In this respect, we noticed that the alleviation of osteoblast differentiation and calcification of human VSMC was reported in the previous study [17]. Therefore, in this study, we aimed to further demonstrate the effects of osteoblast differentiation and calcification of VSMC in high-glucose condition, clarifying the function and mechanism of LIRA as well as GLP-1 in DM combined with AS.

Herein, the effects of the GLP-1 analogue LIRA on VSMC or vascular calcification in high-glucose condition and the involvement of related signaling pathways were investigated *in vitro* and *in vivo*. Therefore, the prospect and significance of LIRA in the treatment of DM complicated with AS were further clarified.

## 2. Materials and Methods

### 2.1. Construction of the DM Animal Model

All procedures involving animal experimental protocols were approved by the Institutional Animal Care and Use Committees (IACUC) of the first affiliated Hospital of Harbin Medical University and follow the ARRIVE guidelines. Clean Sprague-Dawley (SD) rats (Beijing HFK Bioscience, China, 7 weeks, weight ± 200 g) were randomly divided into groups of control, LIRA, DM + AS, and DM + AS + LIRA (*n* = 30 per group). Among them, the control and LIRA were fed with normal diet and DM + AS and DM + AS + LIRA were fed with high-fat diet. The high-fat feed is composed of 10% lard, 5% egg yolk powder, 5% whole milk powder, 0.1% bile salt, 1% cholesterol, 5%sucrose, and 73.9% basic feed. After feeding for one month, DM + AS and DM + AS + LIRA were injected intraperitoneally with STZ (35 mg/kg, dissolved in precooled 0.01 M, pH = 4.4 sodium citrate buffer) to induce DM, while control and LIRA were injected with citric acid buffer. The blood glucose of the rats was measured on the 7th and 14th days. The model was established when the blood glucose was ≥16.9 mmol/L; otherwise, 20 mg/kg STZ was replenished again until the model was successfully established. In order to prevent fatal hypoglycemia, rats were given 20% glucose orally for one day after being injected with STZ. After successful establishment of the model, the rats of LIRA and DM + AS + LIRA were continued to be given LIRA (Selleck, USA, NN2211, 200 *μ*g/kg, 2 times/day) until the end of the experiment. In the experiment, the mental state, water intake, food intake, and urine volume of rats were observed and blood glucose was monitored regularly. At 0, 2, and 4 months after the establishment of the model, some rats were killed and the medial edge of the thoracic aorta was taken for further correlation detection.

### 2.2. Immunohistochemical (IHC) Staining

After the tissue samples were deparaffinized, repaired, and blocked with citric acid antigen, they were incubated with antibody SM*α*-actin (Abcam, USA, ab7817, 1 : 200) overnight at 4°C. Afterwards, horseradish peroxidase- (HRP-) conjugated secondary antibody IgG (Abcam, USA, ab150077, goat anti-rabbit, 1 : 400) was added to continue incubation for 1 h at 37°C. As soon as the sections develop, they were immersed in deionized water and stained with DAB (Solarbio, China, DA1010) followed by hematoxylin for visualization. All tissues were pictured with microscopic and viewed with ImageScope and CaseViewer.

### 2.3. Hematoxylin-Eosin Staining

Tissue samples were embedded in paraffin and stained with hematoxylin and eosin in turn. Subsequently, the tissue sample was dehydrated with ethanol and xylene and sealed with neutral gum. The staining effect was observed and photographed under a 400x microscope.

### 2.4. Collection of VSMC

SD rats aged 5–8 weeks were anesthetized on the sterile operating table, and the whole thoracic aorta was quickly isolated. Subsequently, the blood vessels were cut into tissue blocks of 1–2 mm size and soaked in T25 bottles (containing 2 mL fetal bovine serum) 30 min. The tissue blocks were placed at the bottom of the DMEM (ThermoFisher, USA) culture flask (containing 15% FBS) and cultured at 37°C in a 5% CO_2_ incubator for 12 h. After a week, a large number of cells distributed around the tissue mass can be subcultured. The calcifying medium contained 10 mM *β*-glycerophosphate (*β*-GP, Beyotime, ST637) and 50 *μ*g/mL ascorbate (Merck, USA, 134-03-2). The obtained VSMC was intervened differently, including control (5.5 mM glucose), high glucose (HG, 25 mM glucose), LIRA (100 nM), HG + LIRA (20 mM), HG + LY294002 (PI3K antagonist, 50 *μ*M, MCE, USA, HY-10108), HG + LY294002 + LIRA, HG + PD98059 (ERK antagonist, 50 *μ*M, MCE, USA, HY-12028), HG + PD98059 + LIRA, and HG + Exe (9-39) (GLP-1 receptor antagonist, 200 nM, MCE, USA, HY-P0264) + LIRA.

### 2.5. Detection of Alkaline Phosphatase (ALP) Vitality

The 100 *μ*L substrate buffer (ALP kit, Sigma, USA, MAK447) and 20 *μ*L samples (5 *μ*g/*μ*L) were added to the 96-well plate and fully shaken, incubated at 37°C for 15 min. After the termination solution of 80 *μ*L reaction was added and oscillated for 1 min, the absorbance at 520 nm was measured by an enzyme-labeling instrument. The ALP activity is defined as 1 unit of 1 mg phenol produced by the interaction of 15 min with a matrix at 37°C per gram of protein.

### 2.6. Western Blotting

RIPA lysate was used to prepare tissue homogenate to extract protein and NP-40 lysate to obtain cell protein. The protein concentration was measured using the BCA protein kit (TaKaRa, Otsu, Japan, T9300A). Protein was degenerated in sodium dodecyl sulfate (SDS) buffer, followed by separating on SDS-polyacrylamide electrophoresis (PAGE) gel using electrophoresis. After that, they were transferred onto polyvinylidene difluoride (PVDF, Millipore, USA, IPVH00010) membrane and incubated with primary antibody actin (Abcam, USA, ab8226, 1 : 400), BAX (Abcam, USA, ab32503, 1 : 200), Bcl-2 (Abcam, USA, ab182858, 1 : 200), caspase-3 (Abcam, USA, ab32351, 1 : 1000), Cbf*α*-1 (Abcam, USA, ab113203,1 : 200), OPN (Abcam, USA, ab228748, 1 : 200), SM-*α* (Abcam, USA, ab7817, 1 : 500), Akt (Abcam, USA, ab8805, 1 : 200), p-Akt (Abcam, USA, ab38449, 1 : 100), ERK1/2 (Abcam, USA, ab184699,1 : 1000), p-ERK1/2 (Abcam, USA, ab278538,1 : 1000), and *β*-actin (Abcam, USA, ab8226, 1 : 1000) overnight at 4°C. Next, they were incubated with horseradish peroxidase- (HRP-) conjugated secondary antibodies IgG (Abcam, USA, ab150077, goat anti-rabbit, 1 : 5000) at room temperature for 45 min. After the membrane was washed in TBST, the blot was visualized by the enhanced chemiluminescence ECL kit (Thermo Fisher Scientific, NY, USA).

### 2.7. Cell Calcification Detection

The fourth generation of VSMC was collected with a density of 1 × 10^5^ cells/mL. After the cells reached 80% fusion, they were cultured without serum for 24 h. After being cultured with different media for 14 days, the cells in each group were stained with alizarin red. The cells were incubated for 30 min at room temperature, washed twice with PBS, and photographed under a microscope.

### 2.8. Analysis of the Cellular Calcium Content

According to the method provided in the literature [18], we used the calcium colorimetric analysis kit (Abcam, USA, ab102505, 1 : 1000) to analyze the cellular calcium content. Then, the operation was carried out according to the protocol of the kit and the OD value was determined at the wavelength of 610 nm.

### 2.9. Statistical Analysis

All the experiments were repeated three times, and all the data were shown as mean ± standard deviation. All data were processed using SPSS version 17.0 (Chicago, USA). *P* < 0.05 was considered to be statistically significant.

## 3. Results

### 3.1. LIRA Inhibits the Osteogenic Transformation of VSMC in the Thoracic Aorta of DM Rats

The DM rat models were established, and the thoracic aorta of DM rats in 0, 2, and 4 months were used to determine the condition of AS. The osteoblast-like alteration of VSMC was determined by the detection of SM*α*-actin, Cbf*α*-1, and OPN. The results of IHC staining (Figure 1(a)) showed that the positive rate of SM*α*-actin expression in the DM + AS group was significantly lower than that in the control group at 2 months and 4 months but the positive rate increased significantly after LIRA administration. Subcutaneous injection of LIRA alone had no effect on the expression of SM*α*-actin in rats. In addition, these results were further detected by immunoblotting (Figure 1(b)). Additionally, the expression of OPN and Cbf*α*-1 in the DM + AS group increased compared with 2 months. The expression of Cbf*α*-1 and OPN in the DM + AS group was significantly higher than that in the control group at 2 months and 4 months, while was decreased after treatment with LIRA. Similarly, subcutaneous injection of LIRA in DM rats alone had no effect on the expression of Cbf*α*-1 and OPN (Figures 1(c) and 1(d)).

### 3.2. LIRA Slows Down the Progression of as in DM Rats by Inhibiting Vascular Calcification

HE staining showed that there was no significant difference in HE staining of the thoracic aorta among the four groups at 0 months. At 2 months, the DM + AS group showed a thickened arterial wall, endothelial cells were slightly protuberant and irregular, and the arrangement of middle fusiform smooth muscle cells was disordered and thickened obviously. Moreover, in the DM + AS + LIRA group, there was no obvious protuberance of intimal cells and no obvious thickening of the media layer and smooth muscle cells are arranged relatively neatly and slightly thickened. At 4 months, the demarcation of each layer of the arterial wall in the DM + AS group was unclear, endothelial cells fell off, intima thickened, cells arranged irregularly, intima thickened obviously, elastic fibers arranged disorderly, light stained foam cells could be seen in the sub intima, and intima protruded to form plaques. At the same time, in the DM + AS+LIRA group, the boundaries of each layer of the arterial wall were relatively clear, intima media thickening was significantly reduced, the arrangement of cells was relatively regular, foam cells were rare, and there was no obvious plaque formation. The results were similar to those *in vitro* that there was no significant change in the thoracic aorta in the LIRA group and control group (Figure 2(a)).

Then, we detected the effect of LIRA on ALP activity, calcification, and osteogenic marker protein *in vivo*. The ALP activity and calcium content of the thoracic aorta in rats could reflect the degree of vascular calcification to some extent. Our results showed that the ALP activity and calcium content of DM + AS rats increased significantly from 0 to 4 month, which indicated that the degree of AS and calcification became stronger with the extension of time. The activity of ALP in the thoracic aorta of rats was detected at 0, 2, and 4 months, showing that the ALP activity in the DM + AS group was the highest. After being treated with LIRA, the ALP activity decreased significantly (Figure 2(b)). Furthermore, the calcium content (Figure 2(c)) was the highest in the DM + AS group and significantly decreased in the DM + AS + LIRA group compared with control. That is to say, LIRA can delay the progression of AS in DM rats by inhibiting the calcification of the thoracic aorta.

### 3.3. LIRA Inhibits the ALP Activity of VSMC through the PI3K/AKT and ERK1/2 MAPK Signaling Pathways

Next, we extracted vascular smooth muscle cells from the thoracic aorta of SD rats to establish an *in vitro* model. Through the cell morphology under the light microscope and the immunofluorescence detection of SM-*α* actin, we confirmed that VSMC was successfully extracted and the purity met the experimental requirements (Figure 3(a)). As illustrated in Figure 3(b), the ALP activity is an indicator of cell calcification. On the one hand, high glucose can promote the increase of ALP. The ALP activity was reduced after administration of LIRA on a high-glucose basis. In addition, the ALP activity was decreased after VSMC were treated with PI3K antagonist LY294002 or ERK1/2 antagonist PD98059. Furthermore, the VSMC were pretreated with HG + Exe (9-39) + LIRA which contributed to the increase in the ALP level in VSMC (Figure 3(b)). The results of phosphorylated AKT (p-AKT, Figure 3(c)) and p-ERK1/2 (Figure 3(d)) protein expression in each group were shown, which revealed that high glucose could significantly increase the expression of p-AKT and p-ERK1/2 in VSMC. These results showed that LIRA can reduce the ALP activity of VSMC induced by high glucose through PI3K and ERK1/2 signaling pathways and this effect was GLP-1 receptor dependent.

### 3.4. LIRA Inhibits the Osteogenic Transformation and Calcification of VSMC under High-Glucose Condition

Firstly, the protein expression of self-labeled protein SM*α*-actin and bone marker OPN and Cbf*α*-1 in VSMC under different environments was detected. The expression of SM*α*-actin in VSMC (Figure 4(a)) was the lowest in the HG group, while the expression of SM*α*-actin increased after LIRA intervention. On the basis of HG and LIRA, the expression of SM*α*-actin was further increased when VSMC were treated with ERK1/2 antagonist PD98059, while the expression of SM*α*-actin was decreased in cells treated with GLP-1 receptor antagonist Exe-9-39. On the other hand, expression of OPN (Figure 4(b)) was the highest in the HG group but decreased significantly after intervention by LIRA. Treatment with PI3K antagonist LY294002 or ERK antagonist PD98059 could reduce the expression of OPN. On the basis of HG and LIRA, the expression of OPN could be increased through treatment with GLP-1 receptor antagonist Exe-9-39. At the same time, the expression of Cbf*α*-1 (Figure 4(c)) in the HG group was significantly increased but decreased after administration of LIRA compared with that in the control group. The VSMC were treated with antagonists PD98059, which could reduce the expression of Cbf*α*-1. On the basis of HG and LIRA, VSMC treated with PD98059 further decreased the expression of Cbf*α*-1. On the contrary, VSMC treated with GLP-1 receptor antagonist Exe-9-39 increased its expression. Interestingly, there was no significant difference in the expression of OPN, Cbf*α*-1, and SM*α*-actin in VSMC between the LIRA group and the control group. That is, LIRA attenuated SM*α*-actin expression and enhanced the expression of OPN and Cbf*α*-1 partly through the inhibition of PI3K/ERK signaling pathway under high-glucose condition.

Then, we determine the calcification of VSMC using alizarin red staining (Figure 4(d)). Compared with the control group, the alizarin red staining was stronger in the HG group and there were some calcified nodules but the staining level decreased after the intervention of LIRA. Meanwhile, LIRA alone had no effect on the alizarin red staining level of VSMC. Our results showed that high glucose could promote the cartilage-like or osteoblast-like transformation of VSMC and eventually lead to calcification, which could be reversed by LIRA.

Collectively, LIRA has the function of inhibiting the transition of VSMC to osteoblast or chondrocyte and the vascular calcification under high-glucose condition, partly via regulating the PI3K/ERK signaling pathway.

## 4. Discussion

Atherosclerosis (AS) is the most common cardiovascular complication of DM. Vascular remodeling is an important component of the development of AS, which is closely related to the pathological changes of VSMC, including proliferation, migration, and apoptosis [3]. Studies indicated that vascular calcification, which was proved to be partially triggered by osteochondrogenic transdifferentiation of VSMC, also played an important role in the development of AS [17]. Therefore, the investigation of the mechanism underlying the calcification of VSMC and the exploration of the inhibitor of VSMC calcification have been considered as a promising strategy for the treatment of AS. Recently, reports demonstrated the critical role of osteogenic transformation of VSMC in atherosclerotic calcification and the glucose metabolism involved in arterial calcification [19]. In our study, both the *in vitro* and *in vivo* experiments showed that the high-glucose environment could induce osteogenic transformation and calcification of VSMC, thus promoting vascular calcification.

GLP-1 and its analogues (such as LIRA) can regulate blood glucose through a variety of signaling pathways, which has been used in the treatment of DM [20]. At present, more and more studies focus on the cardioprotective effect of GLP-1, including the regulation of cardiovascular risk factors and the impact of cardiac function [21]. In this study, we aim to elucidate the potential regulatory effects of LIRA on DM complicated with AS from the aspects of VSMC phenotype regulation.

Actually, the influence of LIRA on functions or phenotypes of VSMC, especially in DM complicated with AS, is relatively rarely investigated. A previous study demonstrated that LIRA attenuated high-glucose-induced abnormal cell migration, proliferation, and apoptosis of VSMC by activating the GLP-1 receptor and inhibiting ERK1/2 and PI3K/Akt signaling pathways [22]. It has been reported that LIRA was delayed AS in ApoE-deficient mice by enhancing AMP-activated protein kinase and cell cycle regulation and inhibiting the proliferation of VSMC [23]. Furthermore, LIRA-inhibited AGEs induced coronary smooth muscle cell phenotypic transition through inhibiting the NF-*κ*B signaling pathway [24]. Otherwise, LIRA can prevent osteoblastic differentiation of VSMC, resulting in the slowing of arterial calcification (Hu, 2016 #26). There was also evidence that LIRA attenuates osteogenic differentiation and calcification of VSMC through GLP-1R and subsequently activation of the PI3K/Akt/mTOR/S6K1 signaling pathway [25]. Herein, the results of our study revealed that, although LIRA intervention alone possesses relatively weak regulatory effects on VSMC calcification, it could significantly attenuate the high-glucose-induced calcification of VSMC, exerting cardioprotective ability. As expected, this phenomenon is GLP-1R dependent and could be partially eliminated by the treatment of GLP-1R antagonists. Therefore, LIRA could be an option for the treatment of DM combined with AS.

On the other hand, the involvement of PI3K/Akt and ERK1/2 signaling pathways in the regulation of VSMC phenotypes especially calcification has been previously elucidated. For example, Ponnusamy et al. indicated that FTI-277 (farnesyl transferase inhibitor) could suppress VSMC calcification through regulating the PI3K/Akt signaling pathway [7]. Recently, it was reported that microRNA-155 is able to attenuate vascular calcification through regulating Akt signaling and inducing apoptosis of VSMC (Li, 2021, #28). Yang et al. proved the participation of the ERK1/2 pathway in the promotion of VSMC calcification by *Porphyromonas gingivalis*-derived outer membrane vesicles (Yang et al., 2016, #29). Herein, we also recognize the PI3K/Akt and ERK1/2 pathway as downstream of LIRA in the regulation of VSMC calcification. LIRA significantly inhibited the high-glucose-induced activation of Akt and ERK1/2 pathways in VSMC. Administration of antagonists of PI3K/Akt or ERK1/2 signaling pathways could partially abolish the protective effects of LIRA on VSMC calcification. There are some literatures about the influence of LIRA on diabetic AS. It has been reported that LIRA reduces AS in T2DM rats by targeting ER-associated macrophage-derived macrovesicle production [14]. LIRA represses AS by regulating inflammatory pathways in ApoE^−/−^ mice [15]. In this study, we identified that LIRA attenuated diabetic AS by regulating calcification of vascular smooth muscle cells via targeting PI3K/Akt and ERK1/2 signaling. Our finding provides new insights into the mechanism by which LIRA regulates diabetic AS by regulating a novel downstream PI3K/Akt and ERK1/2 signaling, presenting the new phenotypes affected by LIRA in diabetic AS. Meanwhile, there were some limitations in the current study. For example, the PI3K/Akt and ERK1/2 signaling may just be two of the downstream pathways of LIRA-mediated diabetic AS and other potential mechanisms should be explored in the model in future studies. In addition, the validation of the LIRA/PI3K/Akt axis and LIRA/ERK1/2 axis should be performed in the rat model in future investigations.

## 5. Conclusion

In this study, we confirmed that the structural and functional changes of VSMC induced by high glucose exert an important role in the process of DM combined with AS *in vivo* and *in vitro*. LIRA, an analogue of GLP-1, can improve the calcification of VSMC induced by high glucose, thus showing the potential of LIRA in treating DM combined with AS. Mechanistically, the intervention of LIRA on the calcification of VSMC in DM combined with AS was mediated by GLP-1R and was closely related to the inhibition of PI3K/AKT and ERK1/2 signaling pathways (Figure 5).

## Figures and Tables

**Figure 1:** LIRA inhibits the osteogenic transformation of VSMC in the thoracic aorta of DM rats. (a) IHC showed the expression of SM*α*-actin in the rat thoracic aorta (400x). In group DM + AS, 0 months vs. 2 months (*P* < 0.01) and 2 months vs. 4 months (*P* < 0.01). In months 2 and months 4, DM + AS vs. control (*P* < 0.01) and DM + AS + LIRA vs. DM + AS (*P* < 0.01); in group DM + AS, 0 months vs. 2 months (*P* < 0.01) and 2 months vs. 4 months (*P* < 0.01). Protein expression of (b) SM*α*-actin, (c) OPN, and (d) Cbf*α*-1. Data were from three independent experiments expressed as mean ± standard deviation. In month 2 and month 4, DM + AS vs. control (*P* < 0.01) and DM + AS + LIRA vs. DM + AS (*P* < 0.01). In group DM + AS, 0 months vs. 2 months (*P* < 0.01) and 2 months vs. 4 months (*P* < 0.01). ^∗^*P* < 0.01 vs. control; ^#^*P* < 0.01 vs. DM + AS.

**Figure 2:** LIRA slows down the progression of AS in DM rats by inhibiting vascular calcification. (a) HE staining of the thoracic aorta showed the effect of LIRA on the progression of AS in DM rats (400x). (b) ALP activity detection in vitro. (c) Calcium content detection. Data were from three independent experiments expressed as mean ± standard deviation. ^∗^*P* < 0.01 vs. control; ^#^*P* < 0.01 vs. DM + AS. In group DM + AS, 0 months vs. 2 months (*P* < 0.01) and 2 months vs. 4 months (*P* < 0.01).

**Figure 3:** LIRA inhibits the ALP activity of VSMC through the PI3K/AKT and ERK1/2 MAPK signaling pathways. (a) Cell identification by the cell morphology under light microscope (100x) and SM*α*-actin immunofluorescence (400x). (b) ALP activity detection. Data from three independent experiments are expressed as mean ± standard deviation; ^∗^*P* < 0.01 vs. control; ^#^*P* < 0.01 vs. HG; ^†^*P* < 0.01 vs. HG + LIRA. (c) Protein expression of phosphorylated Akt in VSMC. (d) Protein expression of phosphorylated ERK1/2 in VSMC. Data from three independent experiments are expressed as mean ± standard deviation; ^∗^*P* < 0.01 vs. control; ^#^*P* < 0.01 vs. HG; ^∗∗^*P* < 0.05, ^†^*P* < 0.01 vs. HG + LIRA.

**Figure 4:** LIRA inhibits the osteogenic transformation and calcification of VSMC under high-glucose condition. Protein expression of (a) SM*α*-actin, (b) OPN, and (c) Cbf*α*-1. Data from three independent experiments are expressed as mean ± standard deviation. ^∗^*P* < 0.01 vs. control; ^#^*P* < 0.01 vs. HG; ^†^*P* < 0.01 vs. HG + LIRA. (d) Calcification of VSMC tested by alizarin red staining (400x). Data from three independent experiments are expressed as mean ± standard deviation; ^∗^*P* < 0.01 vs. control; ^#^*P* < 0.01 vs. HG; ^∗∗^*P* < 0.05, ^†^*P* < 0.01 vs. HG + LIRA.

**Figure 5:** Schematic diagram of the mechanism of protective effect of liraglutide on diabetic atherosclerosis-induced vascular calcification.

## Data Availability

The datasets used during the present study are available from the corresponding author upon reasonable request.

## Abbreviations

DM: Diabetes mellitus
AS: Atherosclerosis
VSMCs: Vascular smooth muscle cells
LIRA: Liraglutide
ALP: Alkaline phosphatase
IHC: Immunohistochemical
HG: High glucose
PI3K: Phosphatidylinositol-4-diphosphate 3-kinase
AKT: Protein kinase B
GLP-1: Glucagon-like peptide-1
GLP-1R: GLP-1 receptor
T2DM: Type 2 diabetes mellitus.
